# Evaluation Technology of Classroom Students' Learning State Based on Deep Learning

**DOI:** 10.1155/2021/6999347

**Published:** 2021-10-19

**Authors:** Lingjing Chen

**Affiliations:** Students' Affairs Division, Yiwu Industrial & Commercial College, Zhejiang, Yiwu 322000, China

## Abstract

Facial features are an effective representation of students' fatigue state, and the eye is more closely related to fatigue state. However, there are three main problems in the existing research: (1) the positioning of the eye is vulnerable to the external environment; (2) the ocular features need to be artificially defined and extracted for state judgment; and (3) although the student fatigue state detection based on convolutional neural network has a high accuracy, it is difficult to apply in the terminal side in real time. In view of the above problems, a method of student fatigue state judgment is proposed which combines face detection and lightweight depth learning technology. First, the AdaBoost algorithm is used to detect the human face from the input images, and the images marked with human face regions are saved to the local folder, which is used as the sample dataset of the open-close judgment part. Second, a novel reconstructed pyramid structure is proposed to improve the MobileNetV2-SSD to improve the accuracy of target detection. Then, the feature enhancement suppression mechanism based on SE-Net module is introduced to effectively improve the feature expression ability. The final experimental results show that, compared with the current commonly used target detection network, the proposed method has better classification ability for eye state and is improved in real-time performance and accuracy.

## 1. Introduction

Teaching activities mainly include teaching and learning, and learners play an important role in education as subjects. Learning status is an important factor that affects and interferes with their learning efficiency and achievement [1–4]. Learning state includes attention state, fatigue state, and emotional state, among which fatigue state can effectively reflect students' performance in class. Through the analysis of students' fatigue state, we can judge whether students are interested in knowledge points and teachers' teaching. Therefore, the study of students' fatigue state has great educational significance and value.

In the study of students' fatigue state, facial features, including eyes, lips, and expressions, are usually selected for analysis. Related studies have proved that although the lips and other parts can be used to judge and analyze fatigue state, the eye has the greatest correlation with fatigue, and its accuracy is higher than that of other parts [5–7]. Although the face detection technology has been developing for decades and there are many research studies on the location and detection of eyes, it is still affected by external environment, such as light, angle, and obstructions. [4, 8]. Assuming that the camera offset angle is too large and the side face is obtained, it is difficult to locate and detect the eyes. In addition, the existence of obstructions such as glasses, hair, and ornaments also brings some difficulties to eye detection. On the other hand, in order to analyze and judge the fatigue state of learners, it is necessary to define some characteristics artificially to obtain their eye state data [5, 9, 10]. Therefore, the research on these key technologies is of great practical significance.

With the continuous development of computer hardware and software technology, digital image processing technology, and artificial intelligence technology, image feature classification based on depth learning technology has become the most popular research direction. As we all know, in recent years, a research upsurge of deep learning has been set off, which covers many aspects such as pronunciation, text, and image. Depth learning has been well applied in image classification and recognition and can effectively avoid the problems of artificial selection of feature extraction [11, 12]. However, there are three main problems in the existing research: (1) the positioning of the eye is vulnerable to the external environment; (2) the ocular features need to be artificially defined and extracted for state judgment; and (3) although the student fatigue state detection based on convolutional neural network has a high accuracy, it is difficult to apply in the terminal side in real time.

In order to solve the above problems, this study attempts to detect students' fatigue state based on face detection and deep target detection network. Unlike the traditional MobileNetV2-SSD, a new reconstruction pyramid structure is proposed to improve it. It can improve the accuracy of target detection and reduce the model parameters and size as much as possible so that it can be applied to intelligent terminals. A feature enhancement and suppression mechanism based on SE-Net module is introduced to effectively improve the feature expression ability.

## 2. Literature Review

At present, the research on fatigue state detection mainly focuses on the field of fatigue driving, while the research on fatigue state in the field of education tends to be theoretical research, and there are few detection technologies that can be realized. As the detection technology of fatigue state in education field is similar to that of fatigue driving, the research and implementation of key technologies can refer to fatigue driving detection [13, 14]. At present, the research on fatigue driving detection at home and abroad adopts subjective detection and objective detection.

Barua et al. [15] realized a drowsiness judgment system based on face and eye detection technology, which analyzed the eye condition based on eyelid distance and curvature data. The characteristic of this system is that it combines the YCbCr skin color model with the fuzzy logic method and is robust to illumination and angle, but the real-time performance of this system is not strong. Resalat and Saba [16] realized the fatigue state judgment of learners in the network learning environment using regular classification based on the two facial features of eyes and lips, but the accuracy was not high. In Monzo et al. [17], the AdaBoost algorithm was used for face detection, and the template matching method was used for eye detection. Then, a rectangular coordinate system was established with the eyeball center as the origin to detect the total number of continuous black pixels in the horizontal and vertical directions and determine the eye-closed state based on the ratio. However, when the learner's fatigue and inattention are detected on this basis, there is a problem that the accuracy rate of fatigue state judgment is not high.

Shalash [18] proposed the theory that the convolutional neural network could automatically obtain the driver fatigue characteristics by learning. This method did not directly send the whole image to the neural network for identification. The training process and running time of the network were shortened, and the accuracy of the network for eye fatigue detection was improved to a certain extent. Wang et al. [19] proposed the AdUAL-STREAM bidirectional convolutional neural network (GP-BCNN), which avoided the gradient dispersion and over-fitting problems caused by the increase in the number of layers of the network, shortened the training time of the network, and obtained better detection accuracy. Zhao et al. [20] focused on the ability of neural network in feature extraction so that the feature extraction ability obtained by neural network on ImageNet dataset was applied to the extraction of eye features, which solved the problem of small eye dataset and enabled the optimal feature vector to be obtained with less data, resulting in high eye recognition rate. Huu et al. [21] proposed a gesture recognition system based on MobilenetV2, which can achieve good performance on small-scale data sets by reusing the features learned in the network through dense connection.

All of the above methods have defects, which can not fully meet the actual needs of fatigue detection in the field of education. To solve the above problems, this paper proposes a method to judge students' fatigue state by combining face detection with lightweight deep learning technology, which overcomes the interference of environmental factors such as light, occlusion, and angle on the eyes to a certain extent and avoids artificial feature extraction operation. The proposed method can improve the accuracy of target detection while minimizing the parameters and size of the model and can be applied to intelligent terminals.

## 3. Method for Judging Fatigue State of Students

This study is mainly based on face detection, combined with depth target detection network to judge students' eye state, so as to judge learners' fatigue state according to the classification results.

### 3.1. Image Preprocessing and Face Detection

The image data set can be obtained by transforming the video, but in order to make the features more obvious, the image is usually preprocessed before the experiment. The processed image will be the input data of the face detection algorithm, so the preprocessing operation focuses on the algorithm design. Because of the large size of the acquired image, it will take time to process the original image directly. In order to accelerate the speed of face detection, firstly, the image is reduced in size according to the given scale. Face detection is implemented by the AdaBoost algorithm [22–24], which involves Haar features. AdaBoost is extracted based on gray scale image, which has certain requirements for image color. Therefore, the next operation is to transform the existing small-scale images from color space to gray space. The last step is histogram equalization, which enlarges the gray difference between foreground and background in the picture by expanding the dynamic range of gray value, so as to enhance the overall contrast of the picture [25]. In this part, the image is preprocessed by three steps: size reduction, gray scale conversion, and histogram equalization, so as to optimize the later experimental results.

Face detection acts on all pictures in the specified position and marks the faces in each picture in turn. On this basis, the pictures of the face area in the marked frame are stored in the specified folder. The flow of face detection is shown in Figure 1.

First, the AdaBoost algorithm is used to train positive and negative data sets [26], and then the weak classifier is obtained, and then the corresponding image weights are adjusted, and the weights of correctly classified images in positive and negative samples are reduced, while those of incorrectly classified images are increased, thus generating new sample distribution. For the newly generated distribution, the weak classifier is trained to form a new weak classifier, and the above process is repeated until *t* weak classifiers are generated. Then, according to the specified weight distribution, all the generated weak classifiers are superimposed to form a strong classifier.

### 3.2. Design of Deep Target Detection Network Model

The eye state judgment is mainly based on the depth target detection network to classify the eye-opening pictures and the eye-closing pictures. First, a large number of sample pictures are collected, normalized, and converted into a specific picture format and input into the network for feature learning. Then, after training, the model is obtained, and the given picture is classified and identified using this model. The framework for eye state judgment is shown in Figure 2.

### 3.3. Improved MobileNetV2-SSD Network Model

Compared with traditional methods, although the depth network can effectively improve the accuracy of target detection, the number of layers of the network is increasing and the parameters are tens of thousands, so it is difficult to apply it to real life. MobileNetV2 is an advanced deep target detection network [27], and its main contribution is the introduction of inverted residual block and linear bottleneck. Inverse residual convolution block is an important unit of MobileNetV2. The MobileNetV2 inverse residual convolution block structure is shown in Figure 3.

MobileNetV2-SSD network is a target detection framework based on lightweight convolutional neural network. The VGG-16 model in traditional SSD network has many parameters [28], which occupies a large storage space and is not conducive to real-time and accurate running on embedded intelligent terminals. Therefore, replacing VGG network in SSD network architecture with MobileNetV2 network not only improves the detection effect of SSD but also improves the detection speed qualitatively. The MobileNetV2-SSD network structure model is shown in Figure 4.

In Figure 4, the input of the network is RGB image with 300 × 300 pixels, which is extracted by MobileNetV2-SSD network features. This model uses six feature layers for eye detection, including target classification and regression of candidate frames.

### 3.4. New Reconstruction Pyramid Model

The advantage of SSD is that it adds pyramid feature layer structure, makes predictions on each layer, and has better adaptability to targets with different sizes. However, SSD has no connection among feature layers and cannot make full use of the local detail features of low-level feature maps and the global semantic features of high-level feature maps. However, the recognition of small objects relies heavily on context information, which leads to low detection rate of eyes.

In order to enhance the detection ability of eye targets and improve the overall detection accuracy of the network, this paper proposes an improvement based on MobileNetV2-SSD, which fuses the shallow detail features extracted by MobileNetV2-SSD with the high-level semantic features to obtain a new feature layer and reconstructs a set of feature pyramids according to the new feature map. In order to make better use of low-level local detail features, this paper also brings 38 × 38 feature maps into the fusion range. The improved MobileNetV-SSD network structure is shown in Figure 5.

### 3.5. Feature Enhancement and Suppression Mechanism Based on SE-Net Module

SE-Net is the abbreviation of squeeze-and-excitement networks [29], which is mainly used to redistribute the weights of each channel to assist the network to learn the most important features. It also suppresses those features which are of little use, improves the expression ability of the network, and enhances the robustness of the model, so that it can also show excellent performance in the face of complex tasks. The overall structure is shown in Figure 6.

In Figure 6, *X* is the input, *U* is the output of each convolution layer of the network, and $\bar{X}$ is the final output after assigning weights. The implementation process of SE-Net module mainly includes three operations: squeeze operation, excitement operation, and fusion operation.

(1) *Squeeze Operation*. In this operation, the input features with the size of *C* × *H* × *W* are synthesized into the feature description of *C* × 1 × 1 by using global pooling, and the calculation formula is as follows:
  (1) $$\begin{array}{c} Z_{c}=F_{sq}\left(u_{c}\right)=\frac{1}{H\times W}\sum_{i=1}^{H}\sum_{j=1}^{W}u_{c}\left(i,j\right), \end{array}$$
where *u*_*c*_ is the output in channel *c*.
(2) *Excitation Operation*. After squeeze, the network only gets a global information, which cannot be used as the weight of channels. Therefore, the dependence relationship between channels is obtained comprehensively through the excitement operation. This operation consists of two fully connected layers and Sigmoid activation function. The formula for this operation is as follows:
  (2) $$\begin{array}{c} S=F_{ex}\left(z,W\right)=\sigma \left(W_{2}\delta \left(W_{1}z\right)\right), \end{array}$$
where *z* is the global information obtained by squeeze operation; *δ* represents ReLU function; and *W*_1_ and *W*_2_ are the weights of two fully connected layers.
(3) *Fusion Operation*. After the abovementioned excitation, the network obtains the weights of each channel of the input feature map *U*, and the rest is to fuse the weights with the original features. The way of fusion is simple multiplication:
  (3) $$\begin{array}{c} \bar{\tilde{X}}=F_{\text{scale}}\left(U_{c},S_{c}\right)=S_{c}\times U_{c}. \end{array}$$

SE-Net is a plug-in module, which can be combined with various basic networks. Therefore, SE-Net is embedded in the network introduced in Section 3.4, and the embedded position is behind the six feature layers participating in prediction. SE-Net embedding diagram is shown in Figure 7.

## 4. Experiment and Analysis

### 4.1. Experimental Environment and Data Set

Deep learning requires higher configuration of computer hardware and software. In order to facilitate the training and testing of the model, this paper chooses to experiment in Linux (Ubuntu14.04) operating system environment. The specific configuration information of the computer is as follows: processor Intel (R) Xeon (R) CPU E5-2630 v3, memory 8G, Window 10 system, and graphics card GTX1080. The training data used in the experiment are a single frame image, so it is necessary to intercept the collected video in a single frame. Because the eyes only occupy a part of the video, directly scaling them to 300 × 300 will affect the feature extraction, so this paper clips the meaningful part of the video before extracting the single frame of the video. The results of eye area location and detection are shown in Figure 8.

### 4.2. Effectiveness Verification of Improved Module

In order to verify the effectiveness of the improved MobileNetV2-SSD model, two improved small modules were tested independently. The input image size of the training and testing data set was unified to 300 × 300 × 3, batch_size = 64, epoch = 32, and the network configuration remained the same. The experimental results are shown in Table 1.

It can be seen from Table 1 that each module can improve the accuracy by 1%∼2%. Pyramid reconstruction can fuse the shallow feature information and the high-level semantic information, which makes the network better extract the target features, which is beneficial to improve the target detection accuracy. SE-Net sets different weights for the features of different channels, which enhances the weights of feature layers that play a role in eye recognition and improves the classification accuracy.

### 4.3. Performance Test

In order to test the performance and efficiency of the model, this paper analyzes the fatigue state of 10 groups of video files. The video is taken from the learning process of several students in the laboratory under normal and fatigue conditions. Cut out each video, and select the segment with a duration of about 1 min as the experimental material. The test results are shown in Table 2.

The results show that, except for the 10th group, the normal state was misjudged as fatigue state, and all the other experimental groups were judged correctly, indicating that the model has basically met the students' fatigue state detection requirements.

To illustrate the effectiveness of the improved model for student video detection, it is compared with the original MobileNetV2-SSD network. Four typical videos are selected from the data set. One frame is extracted from the student video every 10 frames and input to these two networks for fatigue state detection experiment. The model test results are shown in Figure 9.

It can be seen that the proposed model can provide enough context information for eye detection by using pyramid reconstruction and multilayer feature fusion, so it can better detect eye regions. At the same time, the added SE-Net module also enhances the useful features for fatigue state identification, which reduces the target detection time and greatly improves the detection rate.

## 5. Conclusions

In this paper, based on the traditional MobilenetV2 network structure, an improved MobilenetV2-SSD fatigue detection network model is proposed. The design idea is as follows: first, a new reconstruction pyramid structure is proposed to improve the detection accuracy of small smoke targets; second, the SE-Net module is embedded in the confidence branch, which enhances the effective features, suppresses the features with little contribution, and further improves the detection accuracy. Two improved modules of the proposed network model are tested, respectively, which proves the feasibility of the proposed improved scheme. Compared with the commonly used target detection network model, it is found that the proposed network model has better detection effect and detection efficiency. Later, we will test and improve the performance of MobilenetV2-SSD network model in a larger video data set and analyze the detection effect of large-size image clipping.

## Figures and Tables

**Figure 1:** Flow of face detection.

**Figure 2:** Framework for eye state judgment.

**Figure 3:** MobileNetV2 inverse residual convolution block structure.

**Figure 4:** MobileNetV2-SSD network structure model.

**Figure 5:** The improved MobileNetV-SSD network structure.

**Figure 6:** SE-Net structure diagram.

**Figure 7:** Schematic diagram of SE-NET embedding.

**Figure 8:** The results of eye area location and detection: (a) eye positioning; (b) normal; (c) fatigue.

**Figure 9:** Model test results: (a) test frame number; (b) detection rate.

**Table 1:** Influence of each module on network.

Model	Pyramid reconstruction	SE-Net	Accuracy rate (%)
Mobile Net V 2-SSD 1			94.6
Mobile Net V 2-SSD 2	√		95.3
Mobile Net V 2-SSD 3		√	95.7
Our improved Mobile Net V 2-SSD	√	√	96.8

**Table 2:** Fatigue state detection results.

Sequence number	Types	Number of open-eyed pictures	Number of closed-eye pictures	Open detection number	Closed eyes detection number	Result
1	Fatigue	394	1082	228	1069	Fatigue
2	Normal	1215	285	1072	227	Normal
3	Normal	1055	472	974	395	Normal
4	Fatigue	767	720	721	389	Fatigue
5	Normal	1226	231	1112	156	Normal
6	Fatigue	555	792	456	742	Fatigue
7	Normal	1315	185	1221	112	Normal
8	Fatigue	149	1351	34	1280	Fatigue
9	Normal	724	216	628	196	Normal
10	Normal	946	523	831	476	Fatigue

## Data Availability

The experimental data used to support the findings of this study are available from the corresponding author upon request.
